The article "Ovarian sex cord stromal tumours: analysis of the clinical and sonographic characteristics of different histopathologic subtypes" was published in 2021. Journal: J Ovarian Res.

# Ovarian sex cord stromal tumours: analysis of the clinical and sonographic characteristics of different histopathologic subtypes

**DOI:** 10.1186/s13048-021-00805-0

**Published:** 2021-04-17

**Authors:** Mei-jiao Jiang, Qian Le, Bo-wen Yang, Fei Yuan, Hui Chen

**Affiliations:** 1 Department of Obstetrics and Gynecology, Ruijin Hospital, Shanghai Jiaotong University School of Medicine, Shanghai, 200025 P.R. China; 2 Department of Pathology, Ruijin Hospital, Shanghai Jiaotong University School of Medicine, Shanghai, 200025 P.R. China

**Keywords:** Ovarian thecoma-fibroma groups, Sertoli-Leydig cell tumours, Ultrasound, Simple rules, ADNEX model

## Abstract

**Background:**

Ovarian sex cord stromal tumours (OSCSTs) are rare ovarian tumours and include different histopathologic subtypes. This study aimed to analyse the clinical and sonographic characteristics of different histopathologic OSCST subtypes.

**Methods:**

A total of 63 patients with surgically proven OSCSTs were enrolled in this retrospective study to analyse their clinical and sonographic features. Ultrasound examinations and predictive models were performed before surgery. The clinical and sonographic findings were compared according to the type of OSCST based on the histopathological diagnosis.

**Results:**

The mean age of 63 patients was 52.17 years (range: 17–78 years). Eighteen patients experienced irregular vaginal bleeding (28.57% 18/63), 7 patients exhibited abnormal body hair (11.11%). 2 patients (3.17%) showed an increased level of CA125, and 25 patients (39.68%, 25/63) showed an increased level of testosterone. Forty-two patients had ovarian thecoma-fibroma groups (OTFGs). Six patients had Sertoli-Leydig cell tumours (S-LCTs), 4 patients had Leydig cell tumours (LCTs), 8 patients had ovarian granulosa cell tumours (OGCTs), 2 patients had ovarian steroid cell tumours, not otherwise specified (OSCTs-NOS), and one patient had sclerosing stromal tumours (SSTs). The mean diameter of the tumour was 47.9 mm (range: 10–258 mm). Forty-seven masses were hypoechoic (74.60%). Twenty-eight masses had posterior echo attenuation, 22 masses exhibited abundant Doppler flow signals (34.92%), and one patient had ascites (1.59%). The diagnostic accuracy of the Simple Rules (SR) and the Assessment of Different NEoplasias in the adneXa (ADNEX) model in distinguishing benign and malignant OSCSTs was 44% (30/63) and 84% (53/63), respectively. The diagnostic accuracy of the SR for OTFGs, S-LCTs & LCTs & OSCTs-NOS, OGCTs, and SSTs was 47.6% (20/42), 16.67% (2/12), 100% (8/8), and 0% (0/1), respectively. The diagnostic accuracy of the ADNEX model for OTFGs, S-LCTs & LCTs & OSCTs-NOS, OGCTs, and SSTs was 93% (31/42), 58.33% (7/12), 75% (6/8), and 100% (1/1), respectively.

The article "Ovarian sex cord stromal tumours: analysis of the clinical and sonographic characteristics of different histopathologic subtypes" was published in 2021. Journal: J Ovarian Res.

**Conclusions:**

OSCSTs generally appear as a solid mass on ultrasound. Posterior echo attenuation indicates an OTFG. A solid mass with abundant Doppler flow signals indicates an S-LCT, LCT, OSCT-NOS or OGCT. Current predictive models are not very effective, but symptoms, sonographic features and serum hormones are helpful for diagnosis.

## Background

Ovarian sex cord stromal tumours (OSCSTs) are rare ovarian tumours that account for approximately 8% of primary ovarian tumours [1]. OSCSTs are derived from primitive sex cords or stromal cells and include different histopathologic subtypes with benign and malignant properties [2]. The proportion of benign stromal tumours is 0.5 to 3.7% of all benign ovarian tumours, and malignant types represent 5 to 8% of all malignant ovarian tumours [3], while the majority of malignant tumours present as low-grade disease. However, because the constituent cells of tumours are engaged in ovarian steroid hormone production, patients who have OSCSTs are usually hyperandrogenic or hyperoestrogenic. Therefore, a correct preoperative diagnosis is significant for these patients.

As the main method of examining ovarian tumours, ultrasound has the advantages of minimal radiation damage and a simple operation [4, 5], and the diagnostic accuracy of ultrasound has improved in recent years. Nonetheless, ultrasound images of OSCSTs vary by histopathologic subtypes, and in some histopathologic subtypes of OSCSTs, masses are usually undetectable because the echo of these masses is similar to that of the surrounding ovarian tissue. Moreover, some doctors lack knowledge on OSCSTs because of the rarity of the disease. In addition, the levels of some tumour markers and sex hormones could be abnormal in patients suffering from OSCSTs [6, 7], but these are not specific markers for OSCSTs. Consequently, it is still a challenge to correctly diagnose OSCSTs at present.

This study primarily summarized the clinical and sonographic features of different histopathologic subtypes of OSCSTs and explored possible associations among clinical features, sonographic characteristics, and histopathologic subtypes. Furthermore, the diagnostic efficiency of Simple Rules (SR) and the Assessment of Different NEoplasias in the adneXa (ADNEX) model for OSCSTs was investigated. We also aimed to analyse the clinical and sonographic characteristics of different histopathologic subtypes of OSCST.

## Methods

### Clinical data

In our study, data from 63 patients who were proven to have OSCSTs by postoperative pathological results were collected from Shanghai Ruijin Hospital between June 2017 and May 2020. Clinical information, including cancer antigen 125 (CA125) test results, sex hormone (testosterone (T) and estradiol 2 (E2)) test results, and sonographic results of OSCSTs with different histopathologic types, were analysed and compared. Our study was approved by the Ruijin Hospital, Shanghai Jiaotong University School of Medicine Institutional Ethics Committee with exemption to obtain informed consent from individual patients.

The article "Ovarian sex cord stromal tumours: analysis of the clinical and sonographic characteristics of different histopathologic subtypes" was published in 2021. Journal: J Ovarian Res.

### Ultrasound examination

All 63 patients underwent preoperative ultrasound examinations using iU22 and EPIQ5 ultrasound machines (Philips Health Systems, Bothell, WA, USA) and E10 ultrasound machines (GE Healthcare) with a 7.0–9.0 MHz transvaginal probe and a 3.5 MHz transabdominal probe.

Experienced ultrasonographers in gynaecological ultrasound preoperatively assessed sonographic tumour morphology according to the International Ovarian Tumour Analysis (IOTA) consensus about the terms, definitions, and measurements used to describe the ultrasound features of adnexal tumours in 2000 [8]. Multi-dimensional and multi-angle real-time scans were performed to obtain more information about the masses from ultrasound images.

Colour Doppler flow imaging was performed on each tumour, and the Doppler signal was scored according to the standard established by D. Timmerman et al. [8] as follows: score 1: no colour flow signal detected, score 2: only minimal colour signals detected, score 3: moderate colour signals displayed, and score 4: abundant colour signals detected. Both greyscale and Doppler ultrasound images with typical features were digitally recorded in the hard drive of the system.

### Prediction models

The IOTA SR [9] model contains five ultrasound benign features, namely, a unilocular cyst, the presence of solid components for which the largest solid component is < 7 mm in its largest diameter, acoustic shadows, a smooth multilocular tumour, and no detectable blood flow on Doppler examination, and five malignant features, namely, an irregular solid tumour, ascites, at least four papillary structures, an irregular multilocular solid tumour with the largest diameter of at least 100 mm, and very high colour content on colour Doppler imaging. If one or more M-features were present in the absence of B-features, the mass was classified as malignant, and if one or more B-features were present in the absence of M-features, the mass was classified as benign. If both M-features and B-features were present or if none of the 10 features was present, the SR were inconclusive.

The IOTA ADNEX model [10] contains nine predictors (three clinical and six ultrasound variables): age, serum CA125 level, type of centre (oncology referral centre vs non-oncology centre), maximum diameter of the lesion, maximal diameter of the largest solid part of the lesion, more than 10 cyst locules (yes or no), number of papillary projections (0, 1, 2, 3 or > 3), acoustic shadows (yes or no) and ascites (yes or no). The model is available to all on the IOTA website (https://www.iotagroup.org/iota-models-software/adnex-risk-model). After objectively inputting all predictors, the probability ratios of benign and malignant lesions were determined.

The article "Ovarian sex cord stromal tumours: analysis of the clinical and sonographic characteristics of different histopathologic subtypes" was published in 2021. Journal: J Ovarian Res.

### Pathological examination

The surgical pathological specimens were immediately fixated in 4% formaldehyde and embedded in paraffin. The sectioned slides were stained with haematoxylin-eosin (HE) for histopathological assessment using a light microscope. The excised tissues were histologically examined in the pathology department following the guidelines of the World Health Organization (WHO) for the classification of tumours [2]. Malignant tumours were staged according to the new International Federation of Gynecology and Obstetrics (FIGO) criteria [11].

### Statistical analysis

All of the statistical analyses were performed using SPSS 22.0 (SPSS Inc., Chicago, IL, USA). All collected data are descriptive. The Mann-Whitney U-test was used to analyze the continuous data. *P* < 0.05 was considered a statistically significant difference.

## Results

### Clinical information

The mean age of 63 patients was 52.17 years (range: 17-78 years). The proportion of postmenopausal patients was 57.14% (36/63). Among the 63 patients, 18 experienced irregular vaginal bleeding or irregular menstruation (28.57%), 3 patients experienced abdominal pain (4.76%), and 7 patients exhibited abnormal body hair (11.11%). Of 63 patients who underwent the CA125 test, 2 (3.17%) showed increased levels, with a mean level of 29.58 U/ml (range: 3.9-555.1 U/ml) (normal value: <35 U/ml). All individuals underwent testosterone testing: 25 patients showed increased levels, with a mean level of 1.05 ng/ml (range: 0.01-7.69 ng/ml) (normal range: 0.15-0.51 ng/ml), and the mean E level of 63 patients was 58.46 pg/ml (range: 0-273 pg/ml) (Table 1).

**Table 1:** Clinical features with different histopathologic types

Factors	thecoma-fibroma	thecoma	Cell-rich thecoma	fibroma	S-LCTs (Well differentiated)	S-LCTs (Moderate differentiation)	LCTs	OGCTs	OSCTs-NOS	SSTs
Age	56.6 ± 13.587	58.5 ± 2.121	61.0 ± 4.243	48.1 ± 9.192	33.0± 5.657	24.3± 1.414	56.8 ± 14.142	56.5 ± 0.707	44.5 ± 31.820	25
Postmenopausal status	22(0.73)	2(1.00)	2(1.00)	2(0.25)	0(0.00)	0(0.00)	3(0.75)	4(0.50)	1(0.50)	0(0.00)
Irregular vaginal bleeding/ Irregular menstruation	1(0.03)	1(0.50)	0(0.00)	1(0.13)	3(1.00)	3(1.00)	1(0.25)	6(0.75)	1(0.50)	1(1.00)
Abdominal pain	1(0.03)	0(0.00)	1(0.50)	1(0.13)	0(0.00)	0(0.00)	0(0.00)	0(0.00)	0(0.00)	0(0.00)
Abnormal body hair	0(0.00)	0(0.00)	0(0.00)	0(0.00)	1(0.33)	1(0.33)	3(0.75)	0(0.00)	2(1.00)	0(0.00)
CA125(U/ml)	28.62 ± 69.340	26.80 ± 20.082	12.15 ± 1.061	13.90 ± 8.401	10.57± 3.407	8.97± 7.317	12.20 ± 10.745	83.48± 190.716	11.4± 4.596	17.9
T (ng/mL) 0.15–0.51	0.39 ± 0.219	0.48 ± 0.057	0.29 ± 0.028	0.42 ± 0.074	3.76± 3.180	1.29± 1.054	4.72 ± 2.177	0.89± 0.571	4.0± 1.386	0.48
E2	45,87 ± 55.392	59.50 ± 20.506	16.50 ± 20.506	67.13 ± 43.584	82.00± 67.978	51.67± 15.695	53.75 ± 16.399	95.38± 90.517	53.5± 0.707	132
Total	30	2	2	8	3	3	4	8	2	1

The article "Ovarian sex cord stromal tumours: analysis of the clinical and sonographic characteristics of different histopathologic subtypes" was published in 2021. Journal: J Ovarian Res.

### Pathological results

Among 63 patients, 30 had thecoma-fibromas, 2 had thecomas, 2 had cell-rich thecomas, 8 had fibromas, 6 had Sertoli-Leydig cell tumours (S-LCTs) (3 well-differentiated and 3 moderately differentiated tumours), 4 had Leydig cell tumours (LCTs), 8 had ovarian granulosa cell tumours (OGCTs), 2 s had ovarian steroid cell tumours, not otherwise specified (NOS) (OSCTs-NOS), and one had sclerosing stromal tumours (SSTs) (Table 2).

**Table 2:** Surgery and pathological results

Pathological types	Number of cases
thecoma-fibroma	30
thecoma	2
Cell-rich thecoma	2
fibroma	8
S-LCTs (Well differentiated)	3
S-LCTs (Moderate differentiation)	3
LCTs	4
OGCTs	8
OSCTs-NOS	2
SSTs	1
total	63

### Ultrasound findings

Sonographic findings of the different subtypes of OSCSTs in 63 patients are presented in Table 3. The mean diameter of the tumour was 47.9 mm (range: 10–258 mm). Ovarian thecoma-fibroma groups (OTFGs) generally exhibited solid hypoechoic masses (92.06%, 58/63), and other sonographic findings varied by the histopathologic subtype. In this study, all 63 masses were unilateral, 47 masses were hypoechoic (74.60%), 35 masses were regular (55.56%, 35/63), and 47 masses had clear boundaries (74.60%, 47/63). Twenty-eight masses had posterior echo attenuation, 22 masses presented abundant Doppler flow signals (score 4) (34.92%), 33 patients had fluid in the pouch of Douglas (52.38%), and one patient had ascites (1.59%).

**Table 3:** Sonographic characteristics with different histopathologic types

Ultrasound Factors	thecoma-fibroma	thecoma	Cell-rich thecoma	fibroma	S-LCTs (Well differentiated)	S-LCTs (Moderate differentiation)	LCTs	OGCTs	OSCTs-NOS	SSTs
Location										
unilateral	30(1.00)	2(1.00)	2(1.00)	8(1.00)	3(1.00)	3(1.00)	4(1.00)	8(1.00)	2(1.00)	1(1.00)
Bilateral	0(0.00)	0(0.00)	0(0.00)	0(0.00)	0(0.00)	0(0.00)	0(0.00)	0(0.00)	0(0.00)	0(0.00)
Tumor size (mm)	51.57± 45.342	39.00 ± 35.355	73.50 ± 23.577	24.25 ± 10.899	23.3± 4.163	41.33± 20.984	21.0 ± 9.381	82.8 ± 39.561	27.0 ± 0.00	55
Echogenicity										
Hypoechoic	24(0.80)	2(1.00)	1(0.50)	8(1.00)	1(0.33)	3(1.00)	1(0.25)	4(0.50)	2(1.00)	1(1.00)
Iso-echoic	2(0.07)	0(0.00)	0(0.00)	0(0.00)	2(0.67)	0(0.00)	3(0.75)	4(0.50)	0(0.00)	0(0.00)
Hyperechoic	0(0.00)	0(0.00)	0(0.00)	0(0.00)	0(0.00)	0(0.00)	0(0.00)	0(0.00)	0(0.00)	0(0.00)
Mixed-echoic	4(0.13)	0(0.00)	1(0.50)	0(0.00)	0(0.00)	0(0.00)	0(0.00)	0(0.00)	0(0.00)	0(0.00)
Form										
Irregular	14(0.47)	1(0.50)	2(1.00)	4(0.50)	0(0.00)	2(0.67)	1(0.25)	4(0.50)	0(0.00)	0(0.00)
Regular	16(0.53)	1(0.50)	0(0.00)	4(0.50)	3(1.00)	1(0.33)	3(0.75)	4(0.50)	2(1.00)	1(1.00)
Boundary										
Clear	29(0.97)	1(0.50)	1(0.50)	1(0.13)	1(0.33)	2(0.67)	3(0.75)	7(0.88)	1(0.50)	1(1.00)
Not clear	1(0.03)	1(0.50)	1(0.50)	7(0.87)	2(0.67)	1(0.33)	1(0.25)	1(0.13)	1(0.50)	0(0.00)
Posterior echo attenuation										
Yes	22(0.73)	0(0.00)	0(0.00)	6(0.75)	0(0.00)	0(0.00)	0(0.00)	0(0.00)	0(0.00)	0(0.00)
No	8(0.27)	2(1.00)	2(1.00)	2(0.25)	3(1.00)	3(1.00)	4(1.00)	8(1.00)	2(1.00)	1(1.00)
Doppler flow signal										
Score 1(None)	11(0.37)	0(0.00)	1(0.50)	5(0.63)	0(0.00)	0(0.00)	0(0.00)	0(0.00)	0(0.00)	0(0.00)
Score 2(Minimal)	12(0.40)	0(0.00)	0(0.00)	2(0.25)	0(0.00)	1(0.33)	0(0.00)	1(0.13)	0(0.00)	0(0.00)
Score3(Moderate)	5(0.17)	1(0.50)	0(0.00)	0(0.00)	1(0.33)	0(0.00)	0(0.00)	1(0.13)	0(0.00)	0(0.00)
Score4(Abundant)	2(0.07)	1(0.50)	1(0.50)	1(0.13)	2(0.67)	2(0.67)	4(1.00)	6(0.75)	2(1.00)	1(1.00)
RI	0.55± 0.153	0.49	0.35	0.55 ± 0.101	0.51± 0.050	0.41± 0.085	0.61 ± 0.097	0.54 ± 0.091	0.48 ± 0.057	0.34
Fluid in pouch of Douglas but no ascites (n)										
Yes	18(0.60)	1(0.50)	1(0.50)	4(0.50)	1(0.33)	2(0.67)	2(0.50)	2(0.25)	1(0.50)	1(1.00)
No	12(0.40)	1(0.50)	1(0.50)	4(0.50)	2(0.67)	1(0.33)	2(0.50)	6(0.75)	1(0.50)	0(0.00)
Ascites (n)										
Yes	0(0.00)	0(0.00)	0(0.00)	0(0.00)	0(0.00)	0(0.00)	0(0.00)	1(0.13)	0(0.00)	0(0.00)
No	30(1.00)	2(1.00)	2(1.00)	8(1.00)	3(1.00)	3(1.00)	4(1.00)	7(0.88)	2(1.00)	1(1.00)
Total	30	2	2	8	3	3	4	8	2	1

The article "Ovarian sex cord stromal tumours: analysis of the clinical and sonographic characteristics of different histopathologic subtypes" was published in 2021. Journal: J Ovarian Res.

### Diagnostic efficiency of the SR and the ADNEX model

The diagnostic accuracy of the SR was 44% (30/63) in distinguishing benign and malignant OSCSTs. The diagnostic accuracy of the SR for the different histopathologic subtypes of OSCSTs in this study was as follows: OTFGs, 47.6% (20/42); S-LCTs, LCTs, and OSCTs-NOS, 16.67% (2/12); OGCTs, 100%(8/8); and SSTs, 0%(0/1).

The diagnostic accuracy of the ADNEX model for OSCSTs was 84% (53/63) in differentiating between malignant and benign tumours. The diagnostic accuracy of the ADNEX model for OTFGs, S-LCTs & LCTs & OSCTs-NOS, OGCTs, and SSTs was 93% (31/42), 58.33% (7/12), 75% (6/8), and 100% (1/1), respectively.

## Discussion

OSCSTs include different histopathologic subtypes and are classified into three main categories: pure stromal tumours, pure sex cord tumours, and mixed sex cord stromal tumours. The rarity and overlapping histomorphology of various OSCSTs often contribute to diagnostic difficulties [12]. Ultrasound is generally used to assist the diagnosis. In a previous study [13], two-dimensional ultrasound provided an early diagnosis for patients suspected of having malignant tumours, and colour Doppler ultrasound had high diagnostic value for OSCSTs. Our study shows that OSCSTs usually exhibit isoechoic and hypoechoic solid masses with or without obvious blood flow signals. Generally, some patients with these tumours have an abnormal hormone status. However, sonographic findings can reflect pathological changes, and these clinical and sonographic characteristics are not the same between different OSCST histopathologic subtypes. We discuss these characteristics below.

### OTFGs

In our study, OTFGs included thecoma-fibromas, thecomas, cell-rich thecomas, and fibromas, accounting for 1.0 to 4.0% of all ovarian tumours [14–16], and they were often found in postmenopausal women [14], generally with a good prognosis. A published study [17] showed that the typical sonographic features of OTFGs include adnexal hypoechoic masses with clear borders and acoustic attenuation as well as minimal Doppler flow signals, which is similar to our study. Our study showed that 28 of 42 patients with OTFGs were postmenopausal (66.67%, 28/42) in. Acoustic attenuation may be related to the fibrous components in tumours. In our study, 28 masses had posterior echo attenuation, and all of them were from OTFGs (66.67%, 28/42). Among the OTFGs, the proportion of masses with acoustic attenuation was higher in thecoma-fibromas (73.33%, 22/30) and fibromas (87.5%, 7/8) than in thecomas (0%, 0/2) and cell-rich thecomas (0%, 0/2). This may be associated with the fact that thecoma-fibromas and fibromas have more fibrous components than the others. Generally, the blood flow of OTFGs is not rich if a blood flow signal can be detected. Minimal or moderate Doppler flow signals were detected in 20 tumours (47.62%, 20/42), while 5 tumours (11.62%, 5/42) showed abundant flow signals, and the proportion of masses with abundant flow signals was higher in thecomas (50%, 1/2) and cell-rich thecomas (50%, 1/2) than in thecoma-fibromas (6.67%, 2/30) and fibromas (12.5%, 1/8). In addition, OTFGs are commonly misdiagnosed as uterine leiomyomas (Fig. 1).

**Fig. 1:** **a** hypoechoic mass was observed in the right ovary with posterior echo attenuation by two-dimension ultrasound examination, confirmed thecoma-fibroma finally; **b** Energy Doppler showed the hypoechoic mass was with minimal Doppler signals

Most OTFGs were benign, and the IOTA ADNEX model was helpful for distinguishing between benign and malignant OTFGs, with an accuracy of 93% (39/42). However, the SR was less effective, with a diagnostic accuracy of 47.6% (20/42). The possible reason for this difference was that some masses had both M-features and B-features, and the SR was inconclusive.

The article "Ovarian sex cord stromal tumours: analysis of the clinical and sonographic characteristics of different histopathologic subtypes" was published in 2021. Journal: J Ovarian Res.

### S-LCTs & LCTs & OSCTs-NOS

S-LCTs, LCTs, and OSCTs-NOS are rare. S-LCTs are mixed sex cord stromal tumours, and LCTs are pure sex cord tumours. Together, they account for less than 1% of all ovarian tumours [18]. The proportion of OSCTs-NOS is less than 0.1% of all ovarian neoplasms [19]. A previous study showed that a woman’s age [18], endocrine symptoms and typical ultrasound findings contributed to a correct diagnosis, in accordance with our study.

Among the three types of tumours, most secrete testosterone, and patients gradually develop progressive hirsutism, acne, deepening of the voice, temporal baldness and amenorrhea. In our study, most of these symptoms were present in patients who had the three types of tumours listed above. Furthermore, menorrhagia or irregular uterine bleeding could be present among these patients with these tumours. Seven patients had abnormal body hair, and all of these patients had S-LCTs, LCTs, and OSCTs-NOS (58.33%, 7/12). A 69-year-old woman who had LCTs showed hirsutism, deepening of the voice, temporal baldness and vaginal bleeding in the postmenopausal status. When the tumour was surgically removed, these symptoms were gradually relieved (Fig. 2). The above symptoms were associated with the abnormal secretion of androgen and oestrogen. All patients with S-LCTs, LCTs, and OSCTs-NOS showed increased levels (100%, 12/12), with a mean level of 3.50 ng/ml (range: 0.66–7.69 ng/ml) (normal range: 0.15–0.51 ng/ml).

**Fig. 2:** A 69-year-old woman suffered from LCT. a hirsutism preoperation; b relieved hirsutism gradually after operation

The above three types of tumours appear as adnexal solid masses with clear borders and abundant Doppler flow signals on ultrasound, and they generally exhibit hypoechoic or isoechoic features. Ten masses (S-LCTs, LCTs, and OSCTs-NOS) exhibited abundant Doppler flow signals (score 4) (83.33%, 10/12). In the 69-year-old woman who had LCTs, the mass was small and solid with a clear border and abundant Doppler flow signals (Figs. 3 and 4).

**Fig. 3:** A 69-year-old woman suffered from LCT. **a** A solid mass with clear border was detected in the right ovary by ultrasound examination; **b** CDFI findings showed the mass with abundant doppler flow signals; c Intraoperativel findings showed right ovarian was hard, the surface smooth, having a good mobility

**Fig. 4:** Pathological findings confirmed LCT in the 69-year-old woman’s right ovarian. **a** HE results; **b** the result showed calretinin positive; **c** the result showed inhibin positive; d the result showed CD99 positive

The benign and malignant characteristics of these tumours depend on their degree of differentiation. The accuracy of the IOTA ADNEX model was 58.33%, without a particularly satisfying result. The accuracy of the SR was worse (16.67%). Because they usually have malignant features (irregular solid masses, abundant blood flow signals) in the models, over half of them are regarded as benign tumours. Another reason could be that these tumours are very rare, and the correct diagnosis depends on the pathological results.

The article "Ovarian sex cord stromal tumours: analysis of the clinical and sonographic characteristics of different histopathologic subtypes" was published in 2021. Journal: J Ovarian Res.

### OGCTs

OGCTs are rare sex cord stromal tumours that belong to malignant ovarian tumours, accounting for only 2–3% of all ovarian tumours [20] and less than 5% of all malignant ovarian tumours [21]. Pathologically, OGCTs are classified into two subtypes: adult and juvenile forms, in which the adult type accounts for 95% of all OGCTs [22]. Although OGCTs have a favourable prognosis, an incidence of 25–30% metastasis or recurrence makes them ovarian tumours with low malignant potential [23]. These tumours may require additional chemotherapy after surgical removal [24], particularly in patients with stage II-IV granulosa cell tumours [25]. In our study, there were 8 OGCTs among 63 OSCSTs. The masses were generally larger than the other OSCSTs (mean diameters: 82.8 mm and 47.9 mm; *P* = 0.002 < 0.05). Generally, the ultrasound features of OGCTs are solid, hypoechoic or isoechoic masses, with abundant Doppler flow signals. All 8 OGCTs exhibited Doppler flow signals, 6 exhibited abundant Doppler flow signals (score 4) (75%, 6/8), one exhibited moderate Doppler flow signals (12.5%, 1/8), and one exhibited minimal Doppler flow signals (12.5%, 1/8). In our study, only one patient had ascites among 63 with OSCSTs, and her CA125 level was 555.1 U/ml (normal range: <35 U/ml) (Fig. 5). This could be because the patient had a stage II granulosa cell tumour.

**Fig. 5:** A 63-year-old woman suffered from OGCT. **a** a cystic-solid mass was detected in the right ovary by two-dimension ultrasound examination; **b** the Color Doppler showed the mass with abundant doppler flow signal; **c** the Spectrum Doppler showed the mass with low velocity blood flow; **d** ultrasound detected ascites in the pelvis

In our study, with an accuracy of 75% for the IOTA ADNEX model (6/8), the SR was more effective at distinguishing between OGCTs and other benign ovarian tumours (accuracy 100% (8/8)). The IOTA ADNEX model misdiagnosed 2 relatively young patients among 8 patients with OGCTs, and the ages of the two patients were 37 and 42 years, with a mean age of 56.5 years (range: 37–78 years) among all patients with OGCTs.

The article "Ovarian sex cord stromal tumours: analysis of the clinical and sonographic characteristics of different histopathologic subtypes" was published in 2021. Journal: J Ovarian Res.

### SSTs

SSTs account for 2 to 6% of all ovarian stromal tumours [26]. Patients who have SSTs are always young women. It has been reported that these tumours occur predominantly in the second and third decades of life [27]. Due to the rarity of SSTs, it is not always possible to predict the presence of these tumours preoperatively based on clinical and sonographic findings, but histopathological and immunohistochemical examinations can confirm the diagnosis. SSTs usually have a benign course and entail a very good prognosis with conservative surgical treatment [26]. There was only one patient with SSTs in our study: a 25-year-old woman who visited a doctor due to irregular menstruation, and the maximum diameter of the mass was 55 mm. Regarding the prediction models, we found that the SR was false, and the IOTA ADNEX model was correct.

There are several limitations of the study. First, the small number of some sub-types of OCSCTs could have affected the result. Second, lacking control study design. Further study with prospective design is needed.

## Conclusion

OSCSTs are rare ovarian tumours, and they generally appear as solid masses on ultrasound. Posterior echo attenuation is usually indicative of OTFGs. A solid mass with abundant Doppler flow signals indicates an S-LCT, LCT, OSCT-NOS or OGCT. Hormones are also essential for diagnosis. Current predictive models are not very effective in differentiating between benign and malignant OSCSTs. The patient’s clinical symptoms, typical sonographic features, and serum hormones are helpful for diagnosis, but the final diagnosis depends on pathology.

## Data Availability

There are no shared the data and material for this manuscript.

## Abbreviations

OCSCTs: Ovarian Sex cord stromal tumours
CA125: Cancer antigen 125
T: Testosterone
E2: Estradiol 2
SR: Simple Rules
ADNEX model: Assessment of Different NEoplasias in the adneXa model
HE: Hematoxylin- eosin.
S-LCTs: Sertoli-Leydig cell tumours
LCTs: Leydig cell tumours
OGCTs: Ovarian granulosa cell tumours
OSCTs-NOS: Ovarian steroid cell tumours, not otherwise specified
SSTs: Sclerosing stromal tumours.
OTFGs: Ovarian thecoma-fibroma groups
